# Intubating Laryngeal Mask Airway for Airway Management and Blind Tracheal Intubation Through It From 360° Around a Supine Patient: A Randomized Controlled Clinical Study in a Simulated Prehospital Emergency Scenario

**DOI:** 10.7759/cureus.67831

**Published:** 2024-08-26

**Authors:** Ritu Dahiya, Vigya Goyal, Isha Bijarnia, Avnish Bharadwaj

**Affiliations:** 1 Anaesthesiology, Mahatma Gandhi Medical College and Research Institute, Jaipur, IND; 2 Anaesthesiology, Mahatma Gandhi Medical College and Hospital, Jaipur, IND

**Keywords:** lma-guided endotracheal intubation, prehospital emergency airway management, attempts of insertion, 360° position of insertion, intubating laryngeal mask airway

## Abstract

Introduction

In emergency situations, airway management is often given priority over other treatment methods. The preferred technique for airway management of unconscious patients is endotracheal intubation, which has become the standard of care. Intubation of the trachea not only enables controlled ventilation even for extended periods and in any position but also allows for the removal of tracheal secretions.

Supraglottic airways have several advantages over endotracheal intubation, including faster insertion, less need for neuromuscular blockade, and less hemodynamic instability. They can also be used as a bridge to intubation or as a rescue device when intubation fails or is contraindicated.

The aim of this randomized controlled clinical study is to simulate a prehospital emergency/disaster scenario to evaluate and study the feasibility and effectiveness of the use of intubating laryngeal mask airway (ILMA) for onsite airway management from 360 degrees around the patient’s head as in such situations, there may be limited or no access behind the head of the victim. Such a scenario can be extrapolated to disaster conditions where the victims may be trapped under the rubble following a building collapse /earthquake or are trapped in a vehicular road traffic/ train accident. It may take substantial time for extrication and evacuation of such patients to a hospital and hence it may be life-saving to provide prompt and early onsite airway management from wherever access is possible around the victim.

We believe that the provision of a steel handle integrated with the airway tube may provide an opportunity for successful insertion of the device from 360 degrees around the patient merely by suitably changing the way the handle is gripped, so as to allow a single-handed smooth arc-like movement of the device for insertion, irrespective of the position of the rescuer relative to the patient’s head.

Objectives

Our objective is to study the ease and time of insertion of ILMA, the number of attempts for successful ILMA insertion, and oropharyngeal leak pressure attained from unconventional positions in a supine patient.

Materials and methods

This prospective, randomized, observer-blinded controlled trial included 90 patients undergoing elective surgery under general anesthesia. Patients were randomized using a chit and box system for group allocation. Groups were as follows: Group 1 (n=30) - Investigator standing on the back of the head of the patient (0°); Group 2 (n=30) - Investigator standing on the left side facing the patient (120°); Group 3 (n=30) - Investigator standing on the right side facing the patient (240°). Then ease and time of insertion of ILMA, number of attempts for successful ILMA insertion and oropharyngeal leak pressure were noted, and intergroup comparison was done.

Conclusion

ILMA has proved to be an effective ventilatory device and a suitable conduit for intubation in patients lying in the supine position from a conventional standard position standing behind the head of the patient, as well as non-conventional position, facing the patient at 120° or 240° from the standard position.

## Introduction

Airway management is a critical aspect of anesthesia and emergency medicine, pivotal for ensuring adequate ventilation and oxygenation [1]. The ability to secure and maintain a patent airway is fundamental to patient safety and effective treatment outcomes [2]. Inadequate airway management can lead to severe complications, including hypoxia, brain injury, and death [3,4]. Various devices and techniques have been developed to facilitate airway management, among which the laryngeal mask airway (LMA) has gained prominence due to its ease of use and high success rates. The LMA, introduced by Dr. Archie Brain in 1983, has revolutionized airway management by providing an alternative to endotracheal intubation and face-mask ventilation [5]. The LMA is a supraglottic airway device that sits above the glottis, allowing for spontaneous or controlled ventilation without the need for laryngoscopy [6,7]. Its use has become widespread in both elective and emergency settings, offering advantages such as reduced hemodynamic response to insertion, ease of placement, and lower risk of airway trauma compared to traditional intubation methods [8,9].

The intubating laryngeal mask airway (ILMA), or LMA-Fastrach, was developed to facilitate tracheal intubation while maintaining the benefits of the standard LMA [9,10]. The ILMA features a rigid, anatomically curved airway tube and a handle to aid insertion and manipulation. It allows for blind tracheal intubation through the device, providing a conduit for endotracheal tube placement without the need for direct visualization of the vocal cords [11]. This innovation has made ILMA a valuable tool in difficult airway scenarios, offering a higher success rate of intubation compared to conventional LMA [12,13].

Blind tracheal intubation through the ILMA is performed without direct visualization of the larynx, relying on anatomical landmarks and the design of the ILMA to guide the endotracheal tube into the trachea [14,15]. This technique is particularly useful in situations where visualizing the glottis is challenging or impossible, such as in cases of difficult or failed direct laryngoscopy [16]. Blind intubation through ILMA has been shown to be effective in various clinical settings, including prehospital, emergency, and anesthetic induction environments [16,17].

Despite the advancements in airway management devices, securing a patent airway remains a significant challenge, particularly in patients with difficult airway anatomy, trauma, or other complicating factors [18]. The supine position, commonly used during anesthesia and resuscitation, can further complicate airway management due to restricted access and reduced visibility [19]. Therefore, the development and validation of techniques that allow for effective airway management from any position around a supine patient are crucial for improving patient outcomes [19,20].

The concept of managing the airway from 360° around a supine patient addresses the need for flexibility and accessibility in emergency situations. This approach ensures that healthcare providers can perform airway management procedures regardless of their position relative to the patient, enhancing the speed and efficiency of intervention. The ILMA, with its design and functionality, is particularly suited for this approach, allowing for blind tracheal intubation from various angles around the patient [21,22]. Several studies have evaluated the efficacy and safety of the ILMA for blind tracheal intubation. 

While existing literature provides substantial evidence supporting the use of ILMA for blind tracheal intubation, there is limited research on its effectiveness when used from different positions around a supine patient. This study aims to address this gap by evaluating the success rates and safety of ILMA-facilitated blind intubation from 360° around a supine patient. The findings will contribute to the body of knowledge on flexible airway management techniques and potentially inform clinical practice guidelines for emergency and anesthetic airway management. The primary objective of this randomized controlled clinical study is to compare the success rates of blind tracheal intubation through ILMA from various positions around a supine patient. Secondary objectives include assessing the time required for successful intubation, the ease of use of the ILMA from different positions, and the incidence of complications or adverse events associated with the procedure.

## Materials and methods

Study design

This study was a hospital-based, randomized, controlled clinical study conducted to evaluate the efficacy and safety of the ILMA for airway management and blind tracheal intubation from different positions around a supine patient in a simulated prehospital emergency scenario.

Study setting

The study was carried out in the operation theatres of Mahatma Gandhi Medical College and Hospital, Jaipur, from February 2023 to October 2023. The study protocol was approved by the Institutional Ethics Committee and registered with the Clinical Trials Registry of India (CTRI/2023/02/049657).

Study sampling

Patients were randomly assigned to one of three groups using the chit and box system (Figure 1).

**Figure 1:** Consort diagram

Study sample size

The reference ILMA insertion first attempt success rates i. e. 84%, 100%, and 80% for the Supine group, Rt. Lat. Group and Lt. Lat. group respectively were reported previously [23]. Considering the first attempt success rate of the Supine group (control) and Rt. Lat. Group (intervention), sample size is calculated using the following formula [24]:

n = 2(Zα+Zβ)2/ δ

δ = (p1 − p2)/√ (p [1 − p]), where p = (p1 + p2)/2

where Zα is the critical value of the normal distribution at α (e.g. for a confidence level of 95%, α is 0.05 and the critical value is 1.96), Zβ is the critical value of the normal distribution at β (e.g. for a power of 80%, β is 0.2 and the critical value is 0.84) and p1 and p2 are the sample proportions of the two groups. n in each group = 26.58673353; n in each group ~ 30.

Study groups

Patients were divided into three groups based on the position of the investigator: Group 1 (n=30): Investigator standing at the back of the head of the patient (0° position); Group 2 (n=30): Investigator standing on the left side, facing the patient (120° position); Group 3 (n=30): Investigator standing on the right side, facing the patient (240° position).

Study participants

Participants included adult patients aged 20-55 years, of either sex, undergoing elective surgery under general anesthesia requiring orotracheal intubation, and who consented to participate. Patients classified as ASA grade I or II were included. Exclusion criteria were the presence of major systemic diseases, mouth opening less than 2.5 cm, reflex esophagitis, intraoral growth, symptomatic hiatus hernia, non-fasting status, predicted difficult airway, and thyromental distance less than 6 cm.

Study parameters

The study measured the time required for ILMA insertion, the success rate of blind tracheal intubation, oropharyngeal leak pressure, and time metrics for ILMA insertion and intubation.

Time Required for ILMA Insertion

The duration from the time the ILMA is picked up to the appearance of the capnographic waveform after the first manual breath following ILMA insertion.

Success Rate of ILMA Insertion

The percentage of successful ILMA placements on the first attempt was studied. The outcome of each ILMA insertion attempt as successful or unsuccessful was recorded. The success rate was calculated by dividing the number of successful first-attempt insertions by the total number of insertion attempts.

Success Rate of Blind Tracheal Intubation

The percentage of successful tracheal intubations performed through the ILMA without direct visualization of the vocal cords was evaluated. The outcome of each intubation attempt was recorded as successful or unsuccessful. The success rate was calculated by dividing the number of successful intubations by the total number of intubation attempts.

Oropharyngeal Leak Pressure

The pressure at which air begins to leak around the ILMA cuff during positive pressure ventilation was assessed. The oropharyngeal leak pressure was measured using a manometer attached to the anesthesia circuit. The airway pressure was gradually increased and the pressure at which an audible leak is detected was noted.

Number of Attempts

The number of attempts required to successfully insert the ILMA and perform blind tracheal intubation was calculated. The number of attempts taken for each successful ILMA insertion and tracheal intubation was recorded.

Study procedure

After obtaining clearance from the Institute Ethics Committee and written informed consent, a thorough preoperative examination was performed on the day before surgery. Standard monitors were attached to the patients upon arrival in the operation theatre. Patients were premedicated and induced with general anesthesia. The ILMA was then inserted according to the group assignment. The time required for insertion and intubation was recorded, and successful ventilation was confirmed. In groups 2 and 3, the ILMA was inserted from the left or right side, respectively. Following successful placement and intubation, the ILMA was removed, and the tracheal tube was secured.

Study data

Data collection included recording the time required for ILMA insertion and intubation, oropharyngeal leak pressure, and any complications encountered during the procedure.

Data analysis

Statistical analysis was performed to compare the efficacy and safety of ILMA use between the groups. The time for insertion and intubation, success rates, and complications were analyzed using appropriate statistical methods. Quantitative variables were expressed as mean±SD and qualitative variables as percentages and proportions. Statistical significance was assigned at p-values of less than 0.05.

Ethical consideration

The study was conducted after obtaining approval from the Institute Ethics Committee. Written informed consent was obtained from all participants. The study adhered to ethical principles ensuring patient safety and confidentiality.

## Results

In Table 1, the age distribution among the three groups was not significant (P = 0.16), with the average age ranging between 40 and 50 years. This suggests a homogeneous age distribution, minimizing age-related biases in the study outcomes. Similarly, gender distribution showed a preponderance of females in groups 2 and 3, while group 1 had an equal number of males and females. The majority of patients weighed between 50 and 60 kg, with no significant difference in mean weight among the groups. Height distribution was also similar across the groups. These findings indicate that the physical characteristics of the patients were comparable, ensuring that these variables did not influence the study's primary and secondary outcomes (p>0.05 = not significant). 

**Table 1:** Demographic data yr: year; kg: kilogram; cm: centimeter All values are mean values with standard deviation in brackets unless stated otherwise. p-value >0.05 is not significant.

Category	Group 1	Group 2	Group 3	p-value
Age Distribution (Yr)	42.8 (15.6)	48.9(12.4)	49.2 (15.6)	0.16
Gender Distribution	50% Male, 50% Female	70% Female, 30% Male	70% Female, 30% Male	-
Weight Distribution (Kg)	60.1 (7.7)	59.2 (7.4)	61.6 (7.9)	0.38 (NS)
Height Distribution (cm)	163.4 (3.8)	161.5(4.4)	163.0(3.7)	0.18 (NS)

Figure 2 shows the ease of insertion among the different groups. ILMA insertion was easy in 88/90 patients. Some difficulty was encountered in 2/90 patients (one patient in group 2 and one in group 3).

**Figure 2:** Ease of insertion

In Table 2, oropharyngeal leak pressure of ILMA was measured which was noted to be in a range of 18 to 24 cmH2O. The p-value for all three groups was not significant (p-value = 0.91, using ANOVA). On intergroup comparison, the p-value of groups 1 and 2 is 0.94, that of groups 2 and 3 is 0.66 and that of groups 1 and 3 is 0.77 (all calculated using the paired t-test, p-value >0.05 is not significant).

**Table 2:** Oropharyngeal leak pressure of ILMA SD: standard deviation; ILMA: intubating laryngeal mask airway

	Oropharyngeal leak pressure			
Group	No.	Mean	SD	Range
1	30	20.4	1.7	18 to 24
2	30	20.3	1.5	18 to 23
3	30	20.5	1.6	18 to 24

Figure 3 shows the mean time taken for ILMA insertion. The ILMA insertion was equally rapid in 0°, 120°, and 240° positions within the range of 10 to 20 seconds. There is no significant difference in the mean time taken for ILMA insertion in the three groups as suggested by the p-value i.e. 0.29 (by ANOVA, p-value >0.05 is not significant). On intergroup comparison, the p-value of groups 1 and 2 is 0.07, that of groups 2 and 3 is 0.3 and that of groups 1 and 3 is 0.55 (all calculated using the paired T-test, p-value >0.05 is not significant).

**Figure 3:** Mean time taken in ILMA insertion Bars represent mean of ILMA insertion time with standard deviation in error bars. ILMA: intubating laryngeal mask airway

Figure 4 shows blind tracheal intubation time through ILMA. In the majority of the patients, successful intubation was performed in 10-20 seconds. The p-value is 0.33 (using ANOVA) indicating no significant difference between the three groups. The p-values on Intergroup comparison were 0.22, 0.3, and 0.52 for groups 1 and 2, groups 2 and 3, and groups 1 and 3 respectively (using the paired T-test, p-value >0.05 is not significant).

**Figure 4:** Blind tracheal intubation sec: seconds Bars represent mean blind tracheal intubation time in seconds with error bars showing standard deviation.

## Discussion

This study aimed to evaluate the efficacy and safety of the ILMA for airway management and blind tracheal intubation in a simulated prehospital emergency scenario, comparing different operator positions around a supine patient. The findings contribute to the growing body of evidence supporting the use of ILMA in various clinical settings. Here, we discuss the study results in detail, comparing them with past studies and citing relevant literature to provide a comprehensive analysis.

ILMA insertion was easy in 88 out of 90 patients, with only two patients experiencing some difficulty. This high success rate aligns with previous studies, such as that by Komatsu (2004), who reported an ILMA insertion success rate of over 96% in their study. The comparison of ease of insertion attempts between the groups did not reveal any statistical significance (p > 0.05), reinforcing the device's reliability across different operator positions [25].

We have followed the technique of insertion of ILMA as recommended by the manufacturer for use from behind the head of the patient (group 1). We however have modified the technique of insertion of ILMA for group 2 and group 3 patients. Taking advantage of the design features of ILMA, namely, the steering handle meant for single-handed insertion in the sagittal plane in an arc-like manner provides the basis for modification of the insertion technique and is used in our patients in group 2 and group 3, respectively.

We have modified the grip according to the position of the investigator, maintaining the required path of ILMA while inserting as suggested by the manufacturers, making sure that the limitations of human joint movements range do not come in the way.

We achieved a 100% success rate in ILMA insertion, with 86 patients requiring only one attempt and four patients requiring a second attempt (p = 0.61). This finding corroborates the study by Panwar et al. (2013), who documented high success rates with minimal attempts in their assessment of ILMA efficiency. The results indicate that ILMA is a robust tool for securing airways, even in challenging prehospital scenarios [23].

The mean time taken for ILMA insertion was similar across the three groups (p = 0.29), demonstrating the device's efficiency irrespective of the operator's position. Comparable results were observed in the study by Timmermann et al. (2007), where the average insertion times did not significantly differ across various clinical settings [26]. Successful intubation was achieved within 10-20 seconds for the majority of patients, with no significant difference between the groups (p = 0.33). 

The oropharyngeal leak pressure of ILMA ranged between 18 and 24 cmH2O across all groups, with no significant difference (p = 0.91). The results were comparable to the study by Utahashi et al. (2008) where no significant correlation between oropharyngeal leak pressure for any LMA and any position [27].

The statistical analysis showed no significant difference in the success rates and intubation times among the three groups (p-value = 0.33). This indicates that the ILMA is equally effective for blind tracheal intubation from various angles around a supine patient. The uniformity in intubation success across different positions can be attributed to the design of the ILMA, which facilitates a straightforward intubation pathway, allowing the endotracheal tube to be guided effectively into the trachea without the need for direct visualization. In a study by Komatsu et al. (2004) [25], blind intubation via the ILMA offers a high success rate and a clinically acceptable intubation time even in patients in the lateral position. A study by Deshmukh et al. (2020) showed blind tracheal intubation through ILMA is a possible option for airway management in patients with a semi-rigid cervical collar neck position [28].

Based on the findings of this study, it is recommended that the ILMA be integrated into prehospital emergency protocols due to its high success rate and ease of use for blind tracheal intubation from various positions around a supine patient. This approach can enhance the flexibility and effectiveness of airway management in emergency scenarios, potentially improving patient outcomes by enabling rapid and reliable intubation regardless of the responder's position. The study's implications suggest that ILMA could become a standard tool in emergency medical kits, emphasizing the need for comprehensive training for emergency medical personnel in its use.

However, the study has limitations, including its simulation-based design and the controlled hospital environment, which may not fully replicate real-world emergency conditions. Future research should focus on validating these findings in actual prehospital settings, exploring the ILMA's performance in diverse and challenging environments, and comparing its efficacy with other advanced airway management devices.

## Conclusions

In conclusion, our study demonstrates that the ILMA is an effective tool as a ventilation device as well as a conduit for intubation. It can be used in both standard and non-conventional positions with ease in a patient in the supine position from anywhere around a supine patient.

With the rising incidence of emergency trauma and associated complications of rapid sequence induction, emergency physicians and paramedics may need a rescue airway device that can be quickly inserted from any position and allows for tracheal intubation in restricted access situations. The ILMA shows promise for pre-hospital emergency airway management with a relatively short learning curve. By making slight adjustments to the grip, it can be effectively used for prompt airway intervention in trapped victims, whether they are lying horizontally under rubble.

## References

[1] Avva U, Lata JM, Kiel J (2024). Airway management. StatPearls [Internet].

[2] Roberts K, Whalley H, Bleetman A (2005). The nasopharyngeal airway: dispelling myths and establishing the facts. Emerg Med J.

[3] Mosier JM, Stolz U, Chiu S, Sakles JC (2012). Difficult airway management in the emergency department: GlideScope videolaryngoscopy compared to direct laryngoscopy. J Emerg Med.

[4] Khan RM, Sharma PK, Kaul N (2011). Airway management in trauma. Indian J Anaesth.

[5] Simon LV, Torp KD (2024). Laryngeal mask airway. StatPearls [Internet].

[6] Lim JA, Jeong MY, Kim JH (2019). Airway management using laryngeal mask airway (LMA) in a patient in a lateral decubitus position: a case report. Medicine (Baltimore).

[7] Strametz R, Bergold MN, Weberschock T (2018). Laryngeal mask airway versus endotracheal tube for percutaneous dilatational tracheostomy in critically ill adults. Cochrane Database Syst Rev.

[8] Singh A, Bhalotra AR, Anand R (2018). A comparative evaluation of ProSeal laryngeal mask airway, I-gel and supreme laryngeal mask airway in adult patients undergoing elective surgery: a randomised trial. Indian J Anaesth.

[9] Armstrong L, Caulkett N, Boysen S, Pearson JM, Knight CG, Windeyer MC (2018). Assessing the efficacy of ventilation of anesthetized neonatal calves using a laryngeal mask airway or mask resuscitator. Front Vet Sci.

[10] Caponas G (2002). Intubating laryngeal mask airway. Anaesth Intensive Care.

[11] Joo HS, Rose DK (1999). The intubating laryngeal mask airway with and without fiberoptic guidance. Anesth Analg.

[12] Reardon RF, Martel M (2001). The intubating laryngeal mask airway: suggestions for use in the emergency department. Acad Emerg Med.

[13] Young B (2003). The intubating laryngeal-mask airway may be an ideal device for airway control in the rural trauma patient. Am J Emerg Med.

[14] El-Emam EM, El Motlb EA (2019). Blind tracheal intubation through the Air-Q intubating laryngeal airway in pediatric patients: reevaluation - a randomized controlled trial. Anesth Essays Res.

[15] Zheng J, Xiao Z, Zhang K, Qiu X, Luo L, Li L (2020). Improved blind tracheal intubation in rats: a simple and secure approach. J Vet Med Sci.

[16] Kleine-Brueggeney M, Nicolet A, Nabecker S, Seiler S, Stucki F, Greif R, Theiler L (2015). Blind intubation of anaesthetised children with supraglottic airway devices AmbuAura-i and Air-Q cannot be recommended: a randomised controlled trial. Eur J Anaesthesiol.

[17] Jagannathan N, Sohn LE, Eidem JM (2013). Use of the air-Q intubating laryngeal airway for rapid-sequence intubation in infants with severe airway obstruction: a case series. Anaesthesia.

[18] Weaver JM (2018). Challenges of airway management. Anesth Prog.

[19] Jarzebowski M, Estime S, Russotto V, Karamchandani K (2022). Challenges and outcomes in airway management outside the operating room. Curr Opin Anaesthesiol.

[20] Karamchandani K, Wheelwright J, Yang AL, Westphal ND, Khanna AK, Myatra SN (2021). Emergency airway management outside the operating room: current evidence and management strategies. Anesth Analg.

[21] Ravindran B (2023). Innovations in the management of the difficult airway: a narrative review. Cureus.

[22] Choi GS, Park SI, Lee EH, Yoon SH (2010). Awake Glidescope® intubation in a patient with a huge and fixed supraglottic mass -a case report-. Korean J Anesthesiol.

[23] Panwar M, Bharadwaj A, Chauhan G, Kalita D (2013). Intubating laryngeal mask airway as an independent ventilatory and intubation device. A comparison between supine, right lateral and left lateral. Korean J Anesthesiol.

[24] Hazra A, Gogtay N (2016). Biostatistics series module 5: determining sample size. Indian J Dermatol.

[25] Komatsu R, Nagata O, Sessler DI, Ozaki M (2004). The intubating laryngeal mask airway facilitates tracheal intubation in the lateral position. Anesth Analg.

[26] Timmermann A, Russo SG, Rosenblatt WH, Eich C, Barwing J, Roessler M, Graf BM (2007). Intubating laryngeal mask airway for difficult out-of-hospital airway management: a prospective evaluation. Br J Anaesth.

[27] Utahashi R (2008). A comparison of airway sealing pressure and positioning of three types of laryngeal mask airway. Showa Univ J Med Sci.

[28] Deshmukh P, Deshmukh D, Dwivedi MB (2020). Comparison of intubation characteristics of McCoy laryngoscope and LMA CTrach with cervical collar in situ: a simulation study. J Evol Med Dent Sci.

